RETRACTED

# Clinical Study on the Efficacy of Microwave Ablation (MA) in the Treatment of Stage I Renal Clear Cell Carcinoma by CT and MRI Imaging

**DOI:** 10.1155/2022/8446294

**Published:** 2022-02-07

**Authors:** Jiang Zhu, Si Chen, Yanchen Wang, TongBin Gao, Yongjian Ji, Shenyang Wang

**Affiliations:** ^1^Weifang Medical University, Weifang 261053, China; ^2^Department of Urology, Weifang People's Hospital, Dezhou 261000, China

## Abstract

We have proposed an effective mechanism to corroborate the efficacy of microwave ablation (MA) in the treatment of stage I renal clear cell carcinoma in this paper. For this purpose, a total of 96 patients with stage I renal clear cell carcinoma presented in our hospital from May 2018 to January 2021 were randomly divided into CT group (*n* = 48) and MRI group (*n* = 48). Patients in both groups were treated with microwave ablation after pathological diagnosis. Patients in the CT group received enhanced CT examination to monitor the therapeutic effect; in contrast, patients in the MRI group received MRI examination to monitor their therapeutic effect. The focus areas before and after tumor microwave ablation were compared between the two groups. The patients were followed up to 1 year after the operation, and the microwave ablation inactivation rates of the two groups were compared according to the postoperative follow-up results. There was no significant difference between CT and MRI in the levels of long and short diameter before and after microwave ablation of renal clear cell carcinoma (*P* > 0.05). In the CT group, CT examination was performed within 24 hours after microwave ablation treatment, and 44 of 48 ablation lesions showed complete ablation. The remaining 4 lesions showed nodular heterogeneous enhancement in the arterial phase, indicating that the tumor remained. Microwave ablation was performed on the residual lesions during the operation, and then enhanced CT was performed again to show that the lesions were ablated completely. In the MRI group, MRI examination was performed within 24 hours after microwave ablation treatment, and 45 of 48 ablation lesions showed complete ablation. The remaining 3 lesions showed nodular heterogeneous enhancement in the arterial phase, indicating that the tumor remained. Microwave ablation was performed on the residual lesions during the operation, and MRI examination showed that the lesions were ablated completely. The patients were followed up to 1 year after the operation, and the microwave ablation inactivation rate of the two groups was compared according to the postoperative follow-up results as the gold standard. The inactivation rate of microwave ablation in the CT group was 89.58 (43/48). The inactivation rate of microwave ablation in the MRI group was 100.00% (48/48). The inactivation rate of microwave ablation in the MRI group was higher than that in the CT group (*χ*^2^ = 5.275, *P* = 0.021).

RETRACTED

## 1. Introduction

Renal tumors account for the highest proportion of primary tumors in the urinary system. Renal cell carcinoma is the most common primary malignant tumor of the kidney, which originates in the tubular epithelial system of the renal parenchyma, accounting for about 23% of all malignant tumors in adults [1, 2]. The common histological types of renal cell carcinoma are renal clear cell carcinoma, renal papillary cell carcinoma, and renal chromophobe cell carcinoma, of which renal clear cell carcinoma accounts for about 65%–80% of renal cell carcinoma [3]. Patients with renal clear cell carcinoma generally have no obvious symptoms in the early stage, and most of them are accidentally found by health examination, and the early detection rate is low. When the tumor increases gradually and forms compression, infiltration, and functional damage to the surrounding tissue structure, it will produce typical symptoms such as abdominal mass, hematuria, and renal pain [4, 5]. Therefore, the early diagnosis of renal cell carcinoma is very important for the choice of operation and prognosis of patients with renal cell carcinoma. In recent years, with the development of medical imaging technology and the improvement of people's health awareness, the early detection rate of renal tumors has significantly increased, and more patients can get early, timely, and effective therapeutics. At present, the treatment of renal clear cell carcinoma is still dominated by traditional radical surgery, including total nephrectomy, partial nephrectomy, and tumor enucleation [6, 7]. However, surgical treatment has the advantages of large trauma, more intraoperative bleeding, and a high incidence of complications, which is not suitable for patients with multiple renal tumors, solitary renal tumors, and metastatic and recurrent renal tumors, unable to tolerate operation and refuse the operation. With the development of medical imaging technology and the continuous progress of microwave ablation technology, percutaneous microwave ablation guided by ultrasound, CT, and MRI has become a new hot spot in the therapeutics of renal tumors. Moreover, how to enhance the body's antitumor immune function and other advantages have been paid more and more attention; this kind of technology is also suitable for stage 1 renal clear cell carcinoma [8–10].

The percutaneous microwave ablation therapy for renal tumor guided by image is that the water-cooled microwave ablation antenna is accurately placed inside the target tumor under the accurate guidance of the imaging equipment. The thermal effect produced by the microwave radiation generator at the end of the microwave ablation antenna renders the central temperature of the tumor tissue to rise rapidly and is gradually transmitted to the surrounding adjacent tissues. Considering that the tumor tissue around the microwave ablation antenna is heated, protein degeneration and cell dehydration occur, which facilitates coagulative necrosis of the tumor tissue [11]. According to the literature, it is reported that there is no significant difference between percutaneous microwave ablation and traditional radical nephrectomy in the treatment of small renal tumors [12]. Percutaneous microwave ablation in the treatment of renal tumors has been widely adopted in the clinic and achieved good therapeutic effect due to its definite curative effect, minimally invasive, simple, easy to protect adjacent organs, and preserving the residual function of the diseased kidney. However, it still has some shortcomings in practical clinical application. The general condition of patients and the experience of operators in clinical work, the limitations of imaging technology, tumor size, shape, location, and adjacent tissues around the tumor will increase the difficulty of treatment in varying degrees and may bring about incomplete tumor ablation and whether the tumor ablation completely directly affects the patient's next treatment plan [13]. Therefore, it is very important to accurately evaluate the efficacy of local microwave ablation.

RETRACTED

At present, according to the literature report, there is no reasonable and unified evaluation standard for the curative effect of microwave ablation of renal tumors. Some scholars establish that the short-term curative effect after microwave ablation therapy is mainly judged by imaging examination of tumor area after treatment and rebiopsy of suspected tumor residual site, but blind puncture biopsy of suspected tumor residual site has great one-sidedness; therefore, in order to ensure a good therapeutic effect and reduce the incidence of incomplete local ablation after microwave ablation, an imaging examination method which can objectively, comprehensively, and accurately evaluate the extent of tumor ablation and the efficacy of local ablation is needed [13]. The commonly used imaging evaluation methods after local microwave ablation of renal tumor include ultrasound, CT, and MRI [14, 15]. Nevertheless, the ultrasound resolution is low, and it is unclear for the small residual tumors after microwave ablation, and the value for monitoring the efficacy of microwave ablation in the treatment of stage I renal clear cell carcinoma is relatively small [16]. Enhanced CT and MRI are noninvasive and relatively accurate means of functional examination, which have a high soft-tissue resolution and can clearly show the shape, location, and adjacent relationship of the tumor [17].

RETRACTED

In this paper, we have proposed an effective mechanism to corroborate the efficacy of microwave ablation (MA) in the treatment of stage I renal clear cell carcinoma. For this purpose, a total of 96 patients with stage I renal clear cell carcinoma presented in our hospital from May 2018 to January 2021 were randomly divided into CT group (*n* = 48) and MRI group (*n* = 48). Patients in both groups were treated with microwave ablation after pathological diagnosis. Patients in the CT group received enhanced CT examination to monitor the therapeutic effect; in contrast, patients in the MRI group received MRI examination to monitor their therapeutic effect. The focus areas before and after tumor microwave ablation were compared between the two groups. The patients were followed up to 1 year after the operation, and the microwave ablation inactivation rates of the two groups were compared according to the postoperative follow-up results.

The rest of the manuscript is arranged according to the following agenda items.

In the subsequent section, the proposed mechanism to evaluate the accuracy of the MA in the treatment of stage 1 renal clear cell carcinoma is presented along with its various possible steps and procedure. In Section 3, experimental results and observations are discussed in detail along with its effectiveness in resolving the issue. General discussion about the proposed mechanism is provided in Section 4 whereas concluding remarks are given in Section 5 of the manuscript which are used to conclude the paper.

## 2. Proposed Method for Measuring Accuracy of MA

### 2.1. General Information

A total of 96 patients with stage I renal clear cell carcinoma treated in our hospital from May 2018 to January 2021 were randomly divided into CT group (*n* = 48) and MRI group (*n* = 48). In the CT group, there were 26 males and 22 females, ranging from 35 to 76 years old, with an average age of (58.32 ± 11.15) years. In the MRI group, there were 25 males and 23 females, ranging from 36 to 76 years old, with an average age of (59.25 ± 11.36) years.

Inclusion criteria are as follows:

1. Patients with renal clear cell carcinoma confirmed by pathological examination are included
2. The tumor stage belongs to stage I, that is, the maximum diameter of the tumor is less than 7 cm, and the scope is limited to the kidney
3. Patients can complete enhanced CT examination, routine MRI examination, and enhanced scan
4. There should be metal implants without MRI taboo, such as aneurysm clip, pacemaker, and artificial heart valve
5. The informed consent form has been signed by the patient and his family

Exclusion criteria are as follows:

1. Those with claustrophobia
2. Those with severe heart, brain, or liver diseases, immune system diseases, or mental or nervous system diseases that cannot be examined
3. Those with severe heart disease, emphysema, asthma, or other reasons unable to hold their breath
4. Contrast agent allergies

RETRACTED

### 2.2. Proposed Treatment Method

Microwave ablation therapeutic instrument and ablation method: using KY-2000 controllable rod temperature wave ablation therapeutic instrument (Nanjing Kangyou Microwave Energy Research Institute), the working frequency is 2450 MHz, the output power is continuously adjustable, and the working modes are continuous and pulse. The microwave ablation therapeutic instrument is connected with the antisticking 14 G water-cooled microwave ablation antenna through a low-loss transmission cable, with a built-in water circulation cooling system, and normal saline circulation cooling is used during microwave ablation treatment to prevent the rod temperature from being too high. In order to improve the accuracy and safety of microwave ablation therapy, there should be fasting for 6 hours before treatment, the establishment of venous passage, intramuscular injection of 30 min to stop bleeding before treatment, ultrasound examination to determine the location, size, number, and surrounding important organ structure of the tumor, routine disinfection of the operation area after determining the puncture point and puncture path, laying aseptic hole towels, and 1% lidocaine after local anesthesia; the skin at the puncture point was cut open for about 2 mm.

Under the guidance of ultrasound, the microwave ablation antenna was placed in the center of the tumor, and after the location was determined, the microwave ablation therapeutic apparatus was turned on for microwave ablation treatment. Different output power (30 w∼50 w), different times (300 s∼800 s), and needle injection times (1 to 3 times) were given according to the size of the focus. After ablation, the microwave ablation antenna was pulled out and the needle was carbonized routinely. The goal of treatment is that the hyperechoic area of the treatment should cover the entire tumor focus together with the renal tissue of 0.5∼1.0 cm around the lesion.

### 2.3. Inspection Method

#### 2.3.1. CT Examination

CT examination was performed within 6 to 24 hours after wave ablation. The DiscoveryCT750 produced by American General Electric Company (GE) was used to examine the patients with routine urological CT scan + enhanced scan. A high-pressure syringe was used to inject a total dose of 60–3.5 ml/s ioferol through the elbow vein at an injection rate of 2.5–80 ml. Cortical and medullary images were obtained at 30–35 s and 70–75 s after injection, respectively. The reconstructed images were 1.25 mm in thickness and 1.25 mm in the interval. The CT images of all patients were saved in JPG.

RETRACTED

#### 2.3.2. MRI Examination

MRI was performed within 6 hours and 24 hours after microwave ablation. The 3.0T SignalExciteHDx superconducting magnetic resonance imaging system produced by GE Company of the United States was used and the abdominal 8-channel phased-array surface coil was used. The patient took the supine position and placed the abdominal 8-channel phased-array surface coil in the front and back of the abdominal wall, and the center was consistent with the midpoint of the xiphoid process and umbilical line. The patients were trained many times to hold their breath at the end of exhalation and achieve the best cooperation after deep breathing. In order to reduce the movement artifacts caused by breathing and the inconsistency of the scanning plane, routine T2WI examination of fat suppressing FSE-XL sequence was performed with 8-channel phased array coil (TR/TE 7059/85.9 ms, 90° flip angle, layer thickness/layer distance 6/2 mm, twice excitation times, twice acquisition times, receiving bandwidth 62.5 kHz FOV 38 cm × 34 cm, matrix 288 × 224). The axial position of breath holding FSPGR sequence was the same as that of inverse biphase T1WI (TR/TE 205/2.5 ms, flip angle 80°, layer thickness/interval 6/2 mm excitation times 0.75 times, acquisition times 0.75 times, receiving bandwidth 62.5 kHz FOV 38 cm × 34 cm, matrix 288 × 200). Axial T1WI enhanced scan (TR/TE185/2.1 ms, flip angle 75°, layer thickness/interval 6/2 mm, excitation times 1, acquisition times 1, accepting bandwidth 62.5 kHz, FOV 38 cm × 34 cm, matrix 384 × 192) of fat suppressing and breath holding FSPGR sequence was performed. The multiphase dynamic contrast-enhanced scan was performed with a 3D-FSPGR (LAVA) sequence, 40 cm 44 slices, and breath holding for 91 s. According to the dose of 0.1 mmol/kg, Gd-DTPA was injected with a magnetic resonance high-pressure syringe at the speed of 1.5∼3 ml/s, and finally, normal saline was injected into the patient about 15 ml to ensure that Gd-DTPA completely entered the patient's body. The cortical scan was performed at 18 seconds after injection of Gd-DTPA, repeated scanning 3 times in the medulla phase (interval between 5 seconds and 10 seconds for each scan), and delayed scanning was performed by 5 min.

RETRACTED

#### 2.3.3. Evaluation Criteria of Therapeutic Effect

According to the evaluation criteria of solid tumors established by WHO, microwave therapy can be divided into

- Complete remission (CR)
- Partial remission (PR)
- Stability (SD)
- Progression (PD)

#### 2.3.4. Evaluation of Target Lesions

CR: all target lesions disappeared. PR: the total length and diameter of baseline lesions were reduced by more than 30%. SD: the sum of the length and diameter of the baseline lesions decreased but did not reach PR or increased but did not reach PD. PD: the maximum diameter and volume of the tumor were larger than that before treatment or new lesions appeared.

### 2.4. Observation Index

The focus areas before and after tumor microwave ablation were compared between the two groups. The patients were followed up to 1 year after the operation, and the microwave ablation inactivation rates of the two groups were compared according to the postoperative follow-up results.

Measurement of lesion size and change before and after microwave ablation: the length, short diameter, and change of the maximum cross section measured by enhanced CT before and after microwave ablation were compared with those measured by MRI before and after ablation. In order to ensure the objectivity and accuracy of the measured values before and after microwave ablation treatment, the slice measurements selected by CT should be consistent with the MRI images as far as possible, with the axial plane showing the largest cross section of the lesions as the standard, and measured and averaged by two experienced ultrasound diagnostic physicians. If there is disagreement on the diagnosis, it is required to reread the film and then record the observation after reaching a consensus on the results of the discussion.

### 2.5. Statistical Analysis

SPSS20.0 statistical software was utilized for statistical analysis. The two examination methods were conducted to evaluate the curative effect of microwave ablation therapy. The *χ*^2^ test of paired four-grid data was used, and the measured value of ablation focus data was expressed as $\bar{x}\pm s$. Paired sample *t*-test was performed on the length, short diameter, and change value of the maximum cross section before and after ablation by the two methods. All the analyses showed that the difference was statistically significant (*P* < 0.05).

## 3. Experimental Results and Observations

In this section, a detailed description and evaluation of the various results obtained through the experiments are presented.

### 3.1. General Clinical Information

There was no significant difference in general clinical information, including sex, age, body mass index, basic medical history, and maximum tumor diameter between the two groups (*P* > 0.05). All the data are presented in Table 1.

RETRACTED

### 3.2. Measurement of Lesion Size before and after Microwave Ablation

There was no significant difference between CT and MRI in the changes of long and short diameter before and after microwave ablation of renal clear cell carcinoma (*P* > 0.05). All the data are presented in Table 2.

### 3.3. Outcome of CT and MRI Examination after Microwave Ablation of Renal Clear Cell Carcinoma

In the CT group, CT examination was performed within 24 hours after microwave ablation treatment, and 44 of 48 ablation lesions showed complete ablation. The remaining 4 lesions showed nodular heterogeneous enhancement in the arterial phase, indicating that the tumor remained. Microwave ablation was performed on the residual lesions during the operation, and then enhanced CT was performed again to show that the lesions were ablated completely. In the MRI group, MRI was performed within 24 hours after microwave ablation treatment, and 45 of 48 ablation lesions showed complete ablation. The remaining 3 lesions showed nodular heterogeneous enhancement in the arterial phase, indicating that the tumor remained. Microwave ablation was performed on the residual lesions during the operation, and MRI examination showed that the lesions were ablated completely.

### 3.4. Comparison of the Efficacy of CT and MRI in the Treatment of Microwave Ablation

The patients were followed up to 1 year after the operation, and the microwave ablation inactivation rate of the two groups was compared according to the postoperative follow-up results as the gold standard. The microwave ablation inactivation rate was 89.58% in the CT group and 100.00% in the MRI group. The inactivation rate of microwave ablation in the MRI group was higher than that in the CT group (*χ*^2^ = 5.275, *P* < 0.01), as shown in Tables 3 and 4.

## 4. Discussion

Renal cell carcinoma remains the most common renal malignant tumor, accounting for more than 80% of renal malignant tumors, ranking seventh and ninth in the incidence of male and female malignant tumors, respectively [18]. The early clinical manifestations of most patients with renal cell carcinoma are often not obvious; when there are hematuria, abdominal pain, and abdominal mass, about 60% of the patients are already in the advanced stage of the disease [19]. The World Health Organization (WHO) formulated the reclassification criteria for renal tumors in 2016. According to the characteristics of cell tissue structure, immunohistochemistry, and genetics, six new renal cell carcinoma subtypes were included in the 2004 renal tumor classification criteria. Among all renal cell carcinoma subtypes, clear cell carcinoma is the most common [20]. At present, traditional surgical radical nephrectomy is still the main treatment of renal tumor, which includes kidney, perirenal fat, perirenal fascia, ipsilateral adrenal gland, and regional enlarged lymph nodes, with a high incidence of complications [21]. In minimally invasive technology, there is a gradual transition from radical nephrectomy to nephron-sparing surgery (NSS) in the treatment of small renal tumors. According to some works of literature, traditional radical nephrectomy and nephron-sparing minimally invasive nephrectomy have a similar therapeutic effect in the treatment of renal tumors, and the latter can retain renal residual function [22]. NSS mainly includes laparoscopic partial nephrectomy (transabdominal or retroperitoneal), tumor enucleation, microwave ablation, radiofrequency ablation, high intensity focused ultrasound, laser ablation, and cryoablation. With the progress of various medical imaging techniques and the continuous improvement of the accuracy of microwave ablation, image-guided percutaneous transhepatic ablation in the treatment of renal tumors has become the most concerned and widely used ablation method owing to its definite curative effect, few complications, repeated treatment, and retention of renal residual renal function [23].

RETRACTED

Percutaneous local microwave ablation of renal tumor is an in situ inactivation technique, whose ultimate goal is to cause complete coagulative necrosis of the whole tumor tissue and reduce the damage of normal renal tissue and surrounding structures [24]. Image-guided percutaneous microwave ablation of renal tumors has been gradually carried out in China, and satisfactory results have been achieved in clinical application. However, in the actual clinical treatment process, the operator's experience, the limitations of imaging technology, the size and shape of the tumor, the location of the tumor, the rich degree of blood supply of the tumor, and the adjacent relationship may affect the therapeutic effect. The extrarenal tumor has a capsule, which is surrounded by retroperitoneal adipose tissue, which can gather the heat generated by microwave in the tumor for a long time, and the curative effect is better. Relatively speaking, the tumor is adjacent to the renal collecting system, ureter, and perirenal vessels, microwave ablation treatment is prone to take away the heat, and affecting the temperature rise may affect the therapeutic effect of the tumor. Whether the tumor is ablated or not directly affects the formulation of the next treatment plan for patients. Therefore, the evaluation of the curative effect after microwave ablation of renal tumors is very important. At present, the ablation effect of renal tumor after microwave ablation is mainly evaluated by imaging examination and puncture biopsy of suspected residual tumor. However, some studies have shown that blind puncture biopsy of suspected sites has a great one-sidedness [25]. Therefore, imaging examination has become the main method to evaluate the curative effect of renal tumors after microwave ablation.

RETRACTED

At present, the clinical methods to evaluate the efficacy of microwave ablation of renal tumor in a short time include contrast-enhanced ultrasound, enhanced CT, or enhanced MRI, in order to understand whether the tumor is ablated completely after microwave ablation [26]. The resolution of ultrasound is low, and it is not clear for the small residual tumors after microwave ablation; thus, it has relatively little value for monitoring the efficacy of microwave ablation in the treatment of stage I renal clear cell carcinoma. CT is a first-line medical imaging means for the diagnosis of renal tumors. Moreover, CT has the advantages of high precision, low cost, noninvasive, and good repeatability. However, some defects encountered in the CT examination of renal clear cell carcinoma may result in important errors. Notably, CT film reading is a subjective work, which depends on the experience of radiologists, and cannot guarantee the reliability between observers and repeatability within observers. MRI examination with a good soft-tissue resolution, the display of minor lesions more clearly, and MRI scan can make a three-dimensional omnidirectional observation of the whole kidney and can accurately show the focus ablation area, perirenal conditions, the occurrence of complications, and so on. At present, there is no reasonable and unified standard for imaging evaluation of ablation efficacy and postoperative follow-up plan after microwave ablation of renal tumor at home and abroad, but they all think that early evaluation is very necessary. Till now, some imaging experts believe that renal tumors should be evaluated by imaging examination within one week after microwave ablation, while other scholars advocate imaging evaluation one month after microwave ablation. If residual tumors are found, supplementary microwave ablation is performed. If no tumor remains or relapses are found, follow-up imaging examination is usually performed 3 months, 6 months, and 1 year after microwave ablation treatment according to the patient's physical condition [27, 28].

Percutaneous microwave ablation is used to treat renal tumors by heating, dehydration, and protein degeneration of tumor tissue, resulting in inactivation of tumor tissue and complete coagulative necrosis of tumor and its surrounding tissues so that the tumor tissue can be completely inactivated in situ [29]. However, in the process of actual clinical treatment, the experience of the operator, the limitation of imaging technology, tumor size and shape, tumor location, and adjacent relationship may make tumor ablation incomplete; therefore, it is very important to accurately evaluate the ablation effect after local microwave ablation. At present, according to the literature report, there is no reasonable and unified evaluation standard for renal tumors after microwave ablation at home and abroad. Some works of literature reported that imaging examination and puncture biopsy of suspected residual tumors are the main methods to judge the curative effect after microwave ablation of renal tumor. However, the blind puncture biopsy of the suspected residual tumor is very one-sided. Therefore, imaging examination plays an important role in the process of microwave ablation, and timely imaging examination during and after operation to determine whether the tumor is ablated completely. If the residual tumor is found to be treated with supplementary microwave ablation in time, it is very important to improve the complete inactivation rate of the tumor.

RETRACTED

Before percutaneous microwave ablation, the size, shape, extent of invasion, adjacent relationship, blood supply, and other information of the tumor can be accurately evaluated by imaging examination, and the treatment plan can be made accordingly. During the treatment, the microwave ablation needle can not only easily and accurately guide the microwave ablation needle to place the target along the preset path but also clearly show the relationship between the microwave ablation needle and the surrounding tissue and the changes of tissue structure in the ablation coagulation area and monitor the whole process of treatment in real time; after treatment, we can not only evaluate whether to achieve the clinical expected effect but also sensitively judge whether there are complications and so on. Through accurate and reliable image guidance, the treatment can not only achieve the purpose of complete coagulative necrosis of the tumor but also minimize the damage to the surrounding tissue structure and the human body, so as to obtain the best effect of local minimally invasive treatment. In this study, CT and MRI were used to monitor the efficacy of microwave ablation in the treatment of stage 1 renal clear cell carcinoma, and its clinical value was discussed.

Since there is no immediate evaluation standard after microwave ablation treatment, timely imaging examination during and after the operation is of great significance to accurately evaluate the ablation effect and guide further treatment, and it is of great significance to improve the detection rate of residual tumors after microwave ablation treatment. Due to the growth characteristics of the tumor, metastasis may occur in the early stage of the tumor. If the ablation range cannot completely cover the tumor, it may result in incomplete ablation. In order to prevent the residual tumor cells around the focus, the ablation range should be beyond the tumor area. According to the literature, it is reported that the appropriate ablation range after microwave ablation of renal tumor is that the ablation area completely covers the tumor and the ablation area reaches the range of peripheral 0.5∼1.0 cm of the tumor [30]. In this study, the ablation area measured by enhanced CT after microwave ablation treatment reached the peripheral range of tumor: long diameter (0.634∼0.912) cm, short diameter (0.647∼0.938) cm; MRI: long diameter (0.623∼0.919) cm, short diameter (0.668∼0.943) m. According to the principle reported in the literature that the range of coagulation and necrosis of renal tumor after microwave ablation should exceed the peripheral 0.5∼1.0 cm of the tumor, the measurement results of CT and MRI showed that the ablation range of the focus was beyond the edge of the tumor area 0.5∼1.0 cm, which conformed to the standard of complete tumor ablation. The results of this study suggest that there is no significant difference between CT and MRI in the changes of long and short diameter before and after microwave ablation of renal clear cell carcinoma. In sum, it is suggested that both of them can accurately evaluate the extent of coagulation and necrosis of renal clear cell carcinoma after microwave ablation.

RETRACTED

In this study, the patients were followed up to 1 year after the operation, and the microwave ablation inactivation rate of the two groups was compared according to the postoperative follow-up results as the gold standard. The inactivation rate of microwave ablation in the CT group was 89.58 (43 ± 48). The inactivation rate of microwave ablation in the MRI group was 100.00% (48/48). The inactivation rate of microwave ablation in the MRI group was higher than that in the CT group (*χ*^2^ = 5.275, *P* = 0.021). Compared to CT checks, the MRI examination can more accurately evaluate the efficacy of microwave ablation in stage I renal clear cell carcinoma. Given that MRI has a good soft-tissue resolution, it can clearly observe the relationship between complete ablation area, residual tumor, and normal renal parenchyma, and MRI has the advantages of multidirectional observation and multiparameter imaging, so it is more accurate in showing the ablation range of lesions and some smaller residual tumors. An MRI examination can make multidirectional and stereoscopic observations of the whole kidney and can accurately judge the efficacy of microwave ablation of renal tumor and the occurrence of complications. It has been reported that MRI is a more accurate imaging method to judge the range of tissue coagulation necrosis after microwave ablation of the renal tumor and has good guidance for accurately judging the curative effect of microwave ablation of renal tumor [31]. However, compared with CT, MRI also has its shortcomings in clinical application. For instance, MRI imaging needed for a long time is not suitable for patients with claustrophobia, and the spatial resolution is relatively low. Moreover, MRI is not suitable for patients with pacemakers, implantation of some metal foreign bodies, artificial heart valves, and aneurysms, and the examination is expensive, so MRI cannot completely replace CT.

In conclusion, both CT and MRI can accurately evaluate the scope of coagulation and a necrotic area of renal tumor after microwave ablation, but MRI can more accurately evaluate the efficacy of microwave ablation of stage I renal clear cell carcinoma than CT. However, MRI also has its shortcomings in clinical application. Therefore, for patients with different conditions, different imaging methods should be adopted to evaluate the detection rate and accuracy of microwave ablation of renal tumors, so as to arrange the treatment plan comprehensively.

## 5. Conclusion

In this paper, we have proposed an effective mechanism to corroborate the efficacy of microwave ablation (MA) in the treatment of stage I renal clear cell carcinoma. For this purpose, a total of 96 patients with stage I renal clear cell carcinoma presented in our hospital from May 2018 to January 2021 were randomly divided into CT group (*n* = 48) and MRI group (*n* = 48). Patients in both groups were treated with microwave ablation after pathological diagnosis. Patients in the CT group received enhanced CT examination to monitor the therapeutic effect; in contrast, patients in the MRI group received MRI examination to monitor their therapeutic effect. The focus areas before and after tumor microwave ablation were compared between the two groups. The patients were followed up to 1 year after the operation, and the microwave ablation inactivation rates of the two groups were compared according to the postoperative follow-up results. Both CT and MRI can accurately evaluate the extent of coagulation and necrosis after microwave ablation of renal tumors, but MRI can more accurately evaluate the efficacy of microwave ablation of stage I renal clear cell carcinoma than CT. However, MRI also has its shortcomings in clinical application. Therefore, for patients with different conditions, different imaging methods should be adopted to evaluate the detection rate and accuracy of microwave ablation of renal tumors, so as to arrange the treatment plan as soon as possible.

RETRACTED

## Figures and Tables

**Table 1:** Comparison of general clinical information of patients [*n* (%), $\bar{x}\pm s\bar{x}$].

Data	*n*	CT group (*n* = 48)	MRI group (*n* = 48)	*χ* ^2^	*P*
Gender					
Male	51	26 (49.25)	25 (32.84)		
Female	45	22 (45.45)	23 (31.82)	0.042	0.838
Age (age)	96	58.32 ± 11.15	59.25 ± 11.36	0.405	0.686
Body mass index (kg/cm^2^)	96	24.82 ± 2.13	25.23 ± 2.35	0.896	0.373
Maximum diameter of tumor (cm)	96	3.83 ± 1.53	3.76 ± 1.56	0.222	0.825
Basic diseases					
High blood pressure					
Yes	36	19 (48.57)	17 (31.43)		
No	60	29 (47.37)	31 (33.68)	0.178	0.673
Type 2 diabetes					
Yes		13 (53.13)	10 (29.69)		
No		35 (45.59)	38 (33.82)	0.515	0.473
Smoking					
Yes		22 (48.76)	21 (32.23)		
No		26 (47.44)	27 (33.33)	0.042	0.838
Drink alcohol					
Yes		28 (49.00)	26 (31.00)		
No		20 (49.00)	22 (31.00)	0.169	0.680

**Table 2:** Measurement of focus range before and after microwave ablation ($\bar{x}\pm s\bar{x}$).

Check method	Cases	Before operation		After operation		Variation value	
		Long diameter (cm)	Short diameter (cm)	Long diameter (cm)	Short diameter (cm)	Long diameter (cm)	Short diameter (cm)
CT	48	3.83 ± 1.53	2.26 ± 1.13	5.56 ± 1.84	3.87 ± 1.37^∗^	1.73 ± 0.34	1.61 ± 0.45
MRI	48	3.76 ± 1.56	2.35 ± 1.52	5.42 ± 1.53	4.13 ± 1.28	1.66 ± 0.28	1.78 ± 0.47
*t*		0.222	−0.329	0.405	−0.961	1.101	−1.810
*P*		0.825	0.743	0.686	0.339	0.274	0.074

**Table 3:** CT evaluation of the efficacy of microwave ablation.

CT check	Follow-up results		Total
	Tumor remnant	Ablation completely	
Tumor remnant	0	0	0
Ablation completely	5	43	48
Total	5	43	48

**Table 4:** MRI evaluation of the efficacy of microwave ablation.

MRI check	Follow-up results			Total
	Tumor remnant		Ablation completely	
Tumor remnant	0	0		0
Ablation completely	0	48		48
Total	0	48		48

## Data Availability

The datasets used and analyzed during the current study are available from the corresponding author upon reasonable request.
